The article "In Vitro Evaluation of the Toxicological Profile and Oxidative Stress of Relevant Diet-Related Advanced Glycation End Products and Related 1,2-Dicarbonyls" was published in 2021. Journal: Oxid Med Cell Longev.

# In Vitro Evaluation of the Toxicological Profile and Oxidative Stress of Relevant Diet-Related Advanced Glycation End Products and Related 1,2-Dicarbonyls

**DOI:** 10.1155/2021/9912240

**Published:** 2021-08-08

**Authors:** Vanesa Cepas, Friederike Manig, Juan C. Mayo, Michael Hellwig, Debora Collotta, Valentina Sanmartino, Rebeca Carrocera-Pumarino, Massimo Collino, Thomas Henle, Rosa M. Sainz

**Affiliations:** ^1^Departamento de Morfología y Biología Celular, Universidad de Oviedo, Spain; ^2^Instituto Universitario de Oncología del Principado de Asturias (IUOPA), Universidad de Oviedo, Instituto de investigación Sanitaria del Principado de Asturias (ISPA), Spain; ^3^Chair of Food Chemistry, Technische Universität Dresden, D-01062 Dresden, Germany; ^4^Institute of Food Chemistry, Technische Universität Braunschweig, Schleinitzstraße 20, D-38106 Braunschweig, Germany; ^5^Department of Neurosciences ‘Rita Levi Montalcini', University of Turin, Italy

## Abstract

During food processing and storage, and in tissues and fluids under physiological conditions, the Maillard reaction occurs. During this reaction, reactive 1,2-dicarbonyl compounds arise as intermediates that undergo further reactions to form advanced glycation end products (AGEs). Diet is the primary source of exogenous AGEs. Endogenously formed AGEs have been proposed as a risk factor in the pathogenesis of diet-related diseases such as diabetes, insulin resistance, cardiovascular diseases, or chronic disease. AGEs may differently contribute to the diet-related exacerbation of oxidative stress, inflammation, and protein modifications. Here, to understand the contribution of each compound, we tested individually, for the first time, the effect of five 1,2-dicarbonyl compounds 3-deoxyglucosone (3-DG), 3-deoxygalactosone (3-DGal), 3,4-dideoxyglucosone-3-ene (3,4-DGE), glyoxal (GO), and methylglyoxal (MGO) and four different glycated amino acids N-*ε*-(carboxyethyl)lysine (CEL), N-*ε*-(carboxymethyl)lysine (CML), methylglyoxal-derived hydroimidazolone-1 (MG-H1), and pyrraline (Pyrr) in a cell line of human keratinocytes (HaCaT). We found that most of the glycated amino acids, i.e., CEL, CML, and MG-H1, did not show any cytotoxicity. At the same time, 1,2-dicarbonyl compounds 3-DGal, 3,4-DGE, GO, and MGO increased the production of reactive oxygen species and induced cell death. MGO induced cell death by apoptosis, whereas 3-DGal and 3,4-DGE induced nuclear translocation of the proinflammatory NF-*κ*B transcription pathway, and the activation of the pyroptosis-related NLRP3 inflammasome cascade. Overall, these results demonstrate the higher toxic impact of 1,2-dicarbonyl compounds on mucosal epithelial cells when compared to glycated amino acids and the selective activation of intracellular signaling pathways involved in the crosstalk mechanisms linking oxidative stress to excessive inflammation.

## 1. Introduction

Advanced glycation end products (AGEs) are a heterogeneous group of molecules formed during the Maillard reaction, which is a spontaneous reaction initiated by a nucleophilic addition between the free amino group of a protein, aminophospholipid, or nucleic acid and the carbonyl group of a saccharide [1, 2]. Protein glycation can occur *in vivo* in tissues and fluids under physiological conditions. It is a slow and continuous process that drives AGE accumulation in tissues during ageing [3]. However, it also takes place *ex vivo*, during food preparation such as baking, cooking, or frying and during storage [4].

Diet is the main exogenous source of AGEs. It has also been described that AGEs are endogenously produced after a high sugar intake, substantially from fructose [5]. In fact, this high fructose consumption generates an increase in AGE levels in tissue and plasma [6, 7].

RAGE (receptor for AGEs) is a multiligand member of the immunoglobulin superfamily of cell surface molecules that, together with AGER1, AGER2, AGER3 receptors, mediates the biological action of AGEs [8]. Nonetheless, some debate persists over the physiological substrate(s) of RAGE and the validity of several poorly characterized AGE-BSA preparations to serve as models for protein-bound AGEs in the body [9, 10]. AGEs-RAGE interaction increases ROS formation [11–14], which initiates several signal transduction cascades involving kinases such as P44/P42 MAPK (ERK1/2), PI3K-AKT or P38 MAPK, and NF-*κ*B activation [15–18]. This leads to the production of inflammatory molecules such as cytokines or chemokines that eventually induce inflammation, apoptosis, and proliferation [19–23]. Furthermore, it has been described that AGEs can activate the NLRP3 inflammasome via oxidative stress and inflammation [24, 25].

There is evidence of an existing relationship between endogenous AGE production, AGEs-RAGE interaction, and chronic hyperglycemia [3, 26, 27]. AGE-induced oxidative stress contributes to the most common diabetes-associated complications such as insulin resistance, atherosclerosis, coronary artery disease, endothelial dysfunction [28], and diabetic nephropathy or retinopathy [29–33].

Upon interaction with RAGE, it has been proposed that AGEs increase oxidative stress. An increase in the intracellular levels of H_2_O_2_, O_2_^•–^, and NO^•^ has been found in endothelial cells [34, 35], macrophages [36], and cardiomyocytes [37]. The elevation of oxidative stress upon interaction with RAGE affects mitochondrial function and cell metabolism in various pathological conditions [38, 39].

One of the main challenges to be confronted is that AGEs are a heterogeneous group of different molecules with different chemical structures, and not all of them might exert the same biological effects. Most of the published studies use glycated albumin or a mixture of different AGEs to investigate their biological activities. Since laboratories usually produce these own compounds, the results are sometimes unreliable and difficult to reproduce. In addition, a more detailed study about the individual cytotoxicity of each compound might be of interest.

To solve these drawbacks, we studied the cytotoxicity of nine different compounds, specifically five 1,2-dicarbonyls: 3-deoxyglucosone (3-DG), 3-deoxygalactosone (3-DGal), 3,4-dideoxyglucosone-3-ene (3,4-DGE), glyoxal (GO), and methylglyoxal (MGO); and four glycated amino acids: N-*ε*-(carboxyethyl)lysine (CEL), N-*ε*-(carboxymethyl)lysine (CML), methylglyoxal-derived hydroimidazolone-1 (MG-H1), and pyrraline (Pyrr) (Figure 1), in a cell model of transformed keratinocytes. The ability to increase oxidative stress, to induce inflammatory pathways, and the type of cell death was investigated.

## 2. Material and Methods

### 2.1. Glycated Amino Acids and 1,2-Dicarbonyls Synthesis

Test substances for cell assays were synthesized as described beforehand: the dicarbonyls 3-deoxyglucosone (3-DG) [40], 3-deoxygalactosone (3-DGal) [40], and 3,4-dideoxyglucosone-3-ene (3,4-DGE) [41] with Z-3,4-DGE being the predominant form and the glycation compounds pyrraline (Pyrr) [42, 43], N-*ε*-(carboxymethyl)lysine (CML) [44], N-*ε*-(carboxyethyl)lysine (CEL) [44], and methylglyoxal-derived hydroimidazolone-1 (MG-H1) [44]. Methylglyoxal (MGO) was obtained from Merck KGaA (Darmstadt, Germany) and glyoxal (GO) from Fisher Sci (Madrid, Spain).

### 2.2. Cell Culture

HaCaT cells (CLS Cell Lines Service) were grown in Dulbecco's Modified Eagle's medium (DMEM) cell culture medium supplemented with 4.5 g/L glucose (Merck KGaA, Darmstadt, Germany), 15 mmol/L 4-(2-hydroxyethyl)-1-piperazineethanesulfonic acid (HEPES) (Merck KGaA, Darmstadt, Germany), 2 mmol/L L-glutamine (Merck KGaA, Darmstadt, Germany), 10% FBS Merck KGaA (Darmstadt, Germany), and 1% antibiotic-antimycotic cocktail (Gibco, Thermo Fisher Scientific, Waltham, MA, USA). Cells were cultured at 37°C in a humidified 5% CO_2_ environment. Cell culture medium was freshly changed every 2 days. Cells were subcultured every 4 days. Briefly, cells were detached using freshly prepared trypsin/EDTA solution (Merck KGaA, Darmstadt, Germany) and incubated at 37°C for 10 minutes. Cells were collected by centrifugation at 300 x g for 5 minutes. Finally, cells were seeded at a split ratio of 1 : 10. To perform the experiments, harvested and centrifuged cells were counted using a Neubauer chamber and seeded in cell culture plates at a density of 2.5 × 10^4^ cells/mL. Cells were always allowed to attach for 48 hours before starting the experiment. Cells were routinely tested for mycoplasma contamination.

### 2.3. Cell Viability Assay by MTT Reduction

To perform the assay, cells were seeded in 96-well plates in 100 *μ*L complete DMEM with 4.5 g/L glucose. After 48 hours, cells were incubated with the different compounds to be tested. After 48 hours incubation, 10 *μ*L 5 mg/mL MTT (Merck KGaA, Darmstadt, Germany) were added to each well and cells were incubated at 37°C and 5% CO_2_ for 4 hours. Then, 100 *μ*L lysis buffer (20% SDS and 50% dimethylformamide, pH 4.7) was added to each well, and cells were left in the incubator at 37°C and 5% CO_2_ overnight [45]. Absorbance was measured at 570 nm *vs.* 690 nm in a Varian Cary 50-MPR UV-Vis spectrophotometer (Agilent Technologies, Santa Clara, CA, USA). Results are shown as the mean of six samples ± SEM.

### 2.4. Cell Viability Assay by Trypan Blue Exclusion

The cell death inhibitors were previously dissolved in 100% dimethyl sulfoxide (DMSO) and then added to culture media from a 1000x stock solution. Therefore, DMSO concentration was never higher than 0.1%, and this concentration was also added to the control group. 2 *μ*mol/L Ferrostatin-1 (0,001% DMSO) (Cayman Chemical, Ann Arbor, MI, USA), 2 mM 3-methyladenine (0,1% DMSO) (Cayman Chemical, Ann Arbor, MI, USA), 100 *μ*mol/L Necrostatin-1 (0,001%) (Cayman Chemical, Ann Arbor, MI, USA), or 10 *μ*M Quinoline-Val-Asp-Difluorophenoxymethyl Ketone (Q-VD-OPh) (0,001% DMSO) (Merck KGaA, Darmstadt, Germany) were employed as inhibitors of ferroptosis, autophagy, necroptosis, and apoptosis, respectively.

To discover the involvement of oxidative stress, 10 mmol/L N-acetyl-cysteine (NAC) (Merck KGaA, Darmstadt, Germany) was used. This compound was freshly dissolved in a culture medium at pH 7.4 and added to the culture media from a 100 mmol/L stock solution. The culture medium was adjusted to the same volume in each group.

To perform the assay, cells were seeded in 24-well plates containing 500 *μ*L complete DMEM with 4.5 g/L glucose. After 48 hours, cells were firstly incubated with the corresponding cell death inhibitor or with NAC for 30 minutes in the incubator at 37°C and 5% CO_2_. Then, the different 1,2-dicarbonyls were added to the culture media. After 48 hours of incubation, cells were detached using trypsin/EDTA solution. Detached and attached cells were collected into the same tube. Cells were stained with 0.4% trypan blue (Merck KGaA, Darmstadt, Germany) using a dilution 1 : 1, allowing the mixture to incubate for 3 minutes at RT. Cells were counted using a Neubauer chamber, and the ratio between viable and nonviable cells was calculated. Results are shown as the mean of three samples ± SEM.

### 2.5. Cell Cycle Analysis

For cell cycle analysis, cells were seeded in 24-well plates in 500 *μ*L complete DMEM with 4.5 g/L glucose. After 48 hours, cells were incubated with the different compounds to be tested. After 48 hours of incubation, cells were detached using trypsin/EDTA solution. Detached and attached cells were added and collected into the same tube. Cells were centrifuged at 300 x g for 5 minutes. Cell pellet was washed twice in PBS and centrifuged at 300 x g for 5 minutes. Cells were then fixed in cold 70% ethanol and left at 4°C for at least 30 minutes. After that, cells were washed once in 2 mL PBS supplemented with 2% bovine serum albumin (BSA) and centrifuged at 300 x g for 5 minutes. Then, the cell pellet was resuspended in 500 *μ*L propidium iodide (PI)/ribonuclease (RNase) Solution (Immunostep S.L, Salamanca, Spain), mixed well, and incubated for 15 minutes at RT. Finally, cells were analyzed in a BD Accuri™ C6 flow cytometer (BD Biosciences, San Jose, CA, USA), and data analysis was performed by using BD Accuri™ C6 Software. At least 10^4^ events per sample were analyzed. Results are shown as the mean of three samples ± SEM.

### 2.6. Quantification of Intracellular and Mitochondrial ROS Levels

To detect intracellular and mitochondrial ROS production, cells were seeded, treated, and collected as described above. To measure O_2_^•-^ production, cells were incubated in 500 *μ*L 5 *μ*mol/L dihydroethidium (DHE) (Bioquochem S.L., Llanera, Spain) for 30 minutes at RT. H_2_O_2_ and HNO_3_^−^ production was examined by incubating cells in 500 *μ*L 5 *μ*mol/L dihydrorhodamine 123 (DHR-123) (Bioquochem S.L, Llanera, Spain) for 30 minutes at RT. To measure mitochondrial O_2_^•-^ production, cells were incubated with 500 *μ*L 5 *μ*mol/L MitoSOX™ Red (Invitrogen, Thermo Fisher Scientific, Waltham, MS, USA) for 10 minutes at 37°C. Finally, cells were analyzed using a BD Accuri™ C6 flow cytometer (BD Biosciences, San Jose, CA, USA), and data analysis was performed using BD Accuri™ C6 Software. At least 10^4^ events per sample were analyzed. Results are shown as the mean of three samples ± SEM.

### 2.7. Annexin-V and 7-AAD Apoptosis Assay

To perform the apoptosis assay, cells were seeded, treated, and collected as described above. Cells were stained using the fluorescein isothiocyanate (FITC) Annexin V Apoptosis Detection Kit with 7-aminoactinomycin D (7-AAD) (Immunostep S.L., Salamanca, Spain) and following the manufacturer's instructions. Briefly, cells were resuspended in 100 *μ*L Annexin V binding buffer. Then, 5 *μ*L Annexin V-FITC and 5 *μ*L 7-AAD were added, and cells were incubated for 15 minutes at RT in the dark. After that, 400 *μ*L Annexin V binding buffer was added to all samples. Finally, cells were analyzed using a BD Accuri™ C6 flow cytometer (BD Biosciences, San Jose, CA, USA), and data analysis was performed using BD Accuri™ C6 Software. At least 10^4^ events per sample were analyzed. To calculate the percentage of apoptotic cells, Annexin V-FITC positive cells as well as Annexin V-FITC- and 7-AAD-positive cells were considered. Results are shown as the mean of three samples ± SEM.

### 2.8. Protein Extraction

For protein extraction, cells were seeded in 100 mm plates containing 10 mL of complete DMEM with 4.5 g/L glucose. After 48 hours, cells were incubated with the different compounds to be tested. After 48 hours of incubation, cells were detached using trypsin/EDTA solution. Detached and attached cells were collected into the same tube. Cells were centrifuged at 300 x g for 5 minutes. Cell pellet was washed twice in PBS and centrifuged at 300 x g for 5 minutes. Then, cells were lysed in radioimmunoprecipitation assay (RIPA) lysis buffer (50 mmol/L Tris-HCl, pH 7.4, 150 mmol/L NaCl, 0.1% sodium dodecyl sulfate (SDS), 1% Igepal C and 0.5% sodium deoxycholate) supplemented with freshly added 2 *μ*g/mL aprotinin, 1 mmol/L dithiothreitol (DTT), 10 *μ*g/mL leupeptin, 1 *μ*g/mL pepstatin, 1 mmol/L phenylmethylsulfonylfluoride (PMSF), 1 mmol/L sodium fluoride, and 200 *μ*mol/L sodium orthovanadate for 30 minutes in ice. After incubation, cells were centrifuged at 15,000 x g for 15 minutes at 4°C, and the supernatant containing the proteins was transferred to a new tube. Proteins were stored at -80°C.

Protein concentration was estimated using the colorimetric Bradford assay [46] (Bioquochem S.L., Llanera, Spain). The absorbance was measured at 595 nm in a Varian Cary 50-MPR UV-Vis spectrophotometer (Agilent, Santa Clara, CA, USA).

### 2.9. Western Blot

To perform western blot assay, 30-50 *μ*g of proteins were mixed 1 : 4 with loading buffer (250 mmol/L Tris-HCl, 40% glycerol, 8% SDS, 0.2% bromophenol blue, and 2.8% *β*-mercaptoethanol). Then, proteins larger than 50 kD were separated in a 10%, and proteins smaller than 50 kD were separated 15% SDS-polyacrylamide gel electrophoresis (PAGE) using a Mini-PROTEAN® Tetra Vertical Electrophoresis Cell (Bio-Rad, Hercules, CA, USA). Then, proteins were electrotransferred to Immobilon®-P polyvinylidene difluoride (PVDF) membranes (Millipore, Merck KGaA, Darmstadt, Germany) using a Mini Trans-Blot® Cell (Bio-Rad, Hercules, CA, USA). After that, the membranes were always stained with Ponceau solution (Bioquochem S.L, Llanera, Spain) to confirm that the proteins were correctly transferred. Then, membranes were incubated with 5% nonfat dry milk in TBS-Tween buffer (TBS-T, Tris-HCl 20 mmol/L, pH 7.4, 150 mmol/L NaCl, 0.05% Tween) for 1 hour at RT. After that, membranes were incubated overnight at 4°C with the corresponding primary antibody anti-*α*-tubulin (1 : 2000, #ab7291, abcam, Cambridge, UK), anti-*β*-actin (1 : 8000, #sc-69879, Santa Cruz Biotechnology, Santa Cruz, CA, USA), anti-catalase (1 : 5000, #219010, Calbiochem, Merck KGaA, Darmstadt, Germany), anti-gasdermin D (1 : 1000, #93709, Cell signaling, Danvers, MS, USA), anti-I*κ*B*α* (1 : 1000, #4814 Cell signaling, Danvers, MS, USA), anti-phospho-I*κ*B*α* (Ser32/36) (1 : 1000, #9246 Cell signaling, Danvers, MS, USA), anti-IKK*β* (1 : 1000, #2370, Cell signaling, Danvers, MS, USA), anti-phospho-IKK*α*/*β* (Ser176/180) (1 : 1000, #2697, Cell signaling, Danvers, MS, USA), anti-NF-*κ*B p65 (1 : 1000, #8242, Cell signaling, Danvers, MS, USA), anti-NLRP3 (1 : 1000, #AG-20B-0014, AdipoGen, Liestal, Switzerland), anti-SOD1 (1 : 5000, #574597, Calbiochem, Merck KGaA, Darmstadt, Germany), and anti-SOD2 (1 : 5000 #06-984, Millipore, Merck, KGaA, Darmstadt, Germany). Primary antibodies were visualized by binding horseradish peroxidase- (HRP-) conjugated anti-rabbit (#12-348, Sigma-Aldrich, Merck KGaA, Darmstadt, Germany), anti-mouse (#12-349, Sigma-Aldrich, Merck KGaA, Darmstadt, Germany), or anti-sheep (#12-342, Sigma-Aldrich, Merck KGaA, Darmstadt, Germany) immunoglobulin G (IgG) secondary antibodies for 1 hour at RT. Antibodies were further detected with Immobilon® Western Chemiluminescent HRP Substrate (Millipore, Merck KGaA, Darmstadt, Germany). Then, an Amersham Hyperfilm™ photographic film (Fisher Scientific, Thermo Fisher Scientific, Waltham, MS, USA) was exposed to the membrane and further developed and fixed in a dark room. Blots were all scanned at 300 dots per inch (dpi) grayscale, and densitometry was quantified by the open-source FIJI software. Results are shown as the mean of 3 samples ± standard error of the mean (SEM).

### 2.10. Statistical Analysis

Unless otherwise indicated, data are presented as mean ± standard error of the mean (SEM). Under normal distribution, differences were estimated using student's *t*-test. When samples did not follow a normal distribution, a nonparametric Mann–Whitney *U* Test was performed. Results were only considered statistically significant if *p* < 0.05. Graphs and statistical analysis were done using the Prism 8 software (GraphPad Software, Inc, USA).

## 3. Results

### 3.1. Most 1,2-Dicarbonyls Were Cytotoxic, whereas Glycated Amino Acids Did Not Alter Cell Viability

As mentioned above, most of the studies published in which the cytotoxicity of AGEs was tested have used albumin glycated by diverse techniques or a solution containing a mixture of different AGEs at unknown concentrations. This, in addition to the many different protocols, makes reproducibility a challenging task. Moreover, to find a relation between the structure and function of these compounds is one of the main aims of this work.

Hence, several synthesized glycated amino acids (CEL, CML, MG-H1, and Pyrr) and 1,2-dicarbonyls (3-DG, 3-DGal, 3,4-DGE, GO, and MGO) were tested on the keratinocyte cell line HaCaT using a wide concentration range to assay their possible cytotoxicity in cell culture. After attachment, cells were incubated for 48 hours with these compounds, and an MTT viability assay was performed.

Only 1,2-dicarbonyls showed cytotoxicity in cell culture (Figure 2(a)). They displayed a clear dose-response, being 3-DGal, GO and MGO significantly cytotoxic compared to the control group above a concentration of 500 *μ*mol/L. When cells were incubated with 3-DGal, the viability of the cells was significantly reduced by 82% at 750 *μ*mol/L. In the case of GO, cell viability was decreased by 59% when tested at a concentration of 1 mmol/L. No surviving cells were found when cultured with 750 *μ*mol/L MGO, and a cytotoxicity of almost 50% with a concentration of 500 *μ*mol/L was observed. The chemically the most reactive dicarbonyl 3,4-DGE was found to be also the most cytotoxic compound. Concentrations of the compound above 50 *μ*mol/L were already significantly cytotoxic, and cell viability after the treatment of the cells with 75 *μ*mol/L 3,4-DGE was dramatically reduced until viability of 11% (Figure 2(b)).

On the other hand, glycated amino acids were much less cytotoxic than 1,2-dicarbonyls, since only Pyrr, at a concentration higher than 500 *μ*mol/L, was able to reduce the viability of HaCaT cells in culture. Thus, 1 mmol/L Pyrr decreased MTT reduction to 61.58%. Although, the cells did not show any signs of cell damage when observed under the microscope. This indicates that Pyrr could affect both proliferation and mitochondrial activity instead of increasing cytotoxicity of HaCaT cells since MTT assay cannot discriminate between them. Interestingly, incubation with CEL, CML, MG-H1, and 3-DG did not show any sign of cell damage (Figure 2(c)). Thus, the following assays addressing individual mechanisms of cytotoxicity were performed only with the dicarbonyl compounds.

### 3.2. GO and MGO Retarded the Cell Cycle in HaCaT Cells

The progression of cell cycle upon incubation with these compounds was assayed to study whether these compounds might reduce cell proliferation and then alter the cell cycle. Thus, cells were incubated with 3-DGal, 3,4-DGE, GO, and MGO for 48 hours, and after that, the cell cycle was studied, staining the cells with PI and, then, analyzing them by flow cytometry. It was found that 3-DGal did not show any change in cell cycle progression compared to control cells. However, 3,4-DGE significantly decreased the number of cells in G_0_/G_1_ phase when compared to the control group. On the other hand, GO and MGO significantly increased the number of cells retained in the S phase, indicating an arrest in the S phase due to activation of the S-phase DNA damage checkpoint (Figure 3).

### 3.3. Antioxidant NAC Recovered 1,2-Dicarbonyl-Mediated Cell Death

It has been proposed that AGEs and their precursors might increase oxidative stress, but this fact was not previously demonstrated with isolated 1,2-dicarbonyl compounds. Consequently, to elucidate whether they were increasing ROS production in this cell culture model and whether cytotoxicity might depend on free radicals, the effect of the antioxidant NAC in preventing cell death induced by these compounds was studied. Thus, cells were preincubated for 30 minutes with 10 mmol/L NAC, and then, the 1,2-dicarbonyls 3-DGal, 3,4-DGE, GO, and MGO were added to the cell culture without removing NAC. After 48 hours of incubation, cell viability was assayed by trypan blue exclusion.

It was found that preincubation with NAC prevented the cytotoxicity of 1,2-dicarbonyls. Upon incubation with 3-DGal and 3,4-DGE, cells showed blebs and irregular borders, an indication for cell damage, which was highly prevented upon coincubation with NAC. Importantly, in the case of MGO incubation, a lot of the cells showed blebs, and cell integrity was completely lost in most cases. Although, when coincubating the cells with NAC, the cell morphology was equal to that observed in the control cells (Figure 4(a)). The role of NAC to prevent the cytotoxicity of 1,2-dicarbonyls was studied by trypan blue exclusion since NAC interferes with formazan, and it cannot be employed in MTT assay. Thus, we found that NAC prevented the cytotoxicity of 1 mmol/L 3-DGal (Figure 4(b)). Similarly, NAC completely prevented the cytotoxicity and recovered cell viability from 84% to 96.97% when cells were treated with 100 *μ*mol/L 3,4-DGE (Figure 4(c)). Interestingly, a reduction of cell viability by GO was not found when trypan blue exclusion was employed, suggesting an effect of the compound on the mitochondrial metabolism of the cells (Figure 4(d)). Finally, the most remarkable result was obtained within the MGO group. Thus, 750 *μ*mol/L MGO treatment reduced the viability of HaCaT cells to an 18.33%. NAC preincubation recovered the viability almost completely to 94% (Figure 4(e)). Altogether, these data account for a feasible role of ROS in mediating 1,2-dicarbonyls cytotoxicity.

### 3.4. 1,2-Dicarbonyls Caused an Increase in ROS and the Production of Antioxidant Enzymes

Then, it was further studied whether 1,2-dicarbonyls triggered ROS production in the human keratinocytes HaCaT cells. Therefore, cells were treated with 3-DGal, 3,4-DGE, GO, and MGO for 48 hours and stained with DHR-123, DHE, and MitoSOX™ Red, and finally analyzed by flow cytometry. Interestingly, individual 1,2-dicarbonyls increased the production of the species measured in HaCaT cells, among the different 1,2-dicarbonyls, GO, and MGO caused a higher ROS production than 3-DGal and 3,4-DGE. Furthermore, superoxide was increased more than twice by MGO than the control group (Figures 5(a)–5(c)).

Because of increasing free radicals' production, cells naturally increase the production of antioxidant enzymes. To evaluate the effect of 1,2-dicarbonyls on the production of antioxidant enzymes as a consequence of the increment of the free radicals produced, cells were incubated with the 1,2-dicarbonyls 3-DGal, GO, and MGO for 48 hours, and the levels of SOD1, SOD2, and catalase were studied by western-blot. In the case of SOD1, only GO significantly increased its levels. However, 3-DGal and GO increased SOD2. The production of CAT did not change after treatment. Besides, since the production of peroxides was increased in the cells upon incubation with 1,2-dicarbonyls, the ratio between catalase and SOD2 production was also studied. Although there was a relative increase in the SOD2/CAT ratio when cells were incubated with 1,2-dicarbonyls, especially GO and MGO, the differences were not statistically significant between groups (Figures 5(d)–5(h)).

### 3.5. MGO Induced Cell Death by Apoptosis in HaCaT Cells

It remains to be determined how 1,2-dicarbonyls lead to cell death and if individual 1,2-dicarbonyls cause cell death by the same mechanism. Therefore, it was firstly assayed whether cells might be dying by apoptosis. To investigate that, cells were incubated with the 1,2-dicarbonyls 3-DG, 3-DGal, 3,4-DGE, GO, and MGO for 48 hours, and after that, they were stained with Annexin-V and 7-AAD and analyzed by flow cytometry.

It was found that the number of apoptotic cells did not change between the control group and cells incubated with 3-DG, 3-DGal, 3,4-DGE, and GO. Outstandingly, the number of cells dying by apoptosis upon MGO incubation was greatly increased, and it reached a mean of 85.35% of the total cells (Figures 6(a) and 6(b)).

To confirm that cells were dying by caspase-mediated apoptosis when incubated with MGO, cells were preincubated with the inhibitor of caspase Q-VD-OPh for 30 minutes, and after that, MGO was added to the cell culture. Cells were incubated with both compounds for 48 hours, and then, cell viability was assayed by trypan blue exclusion. When incubating the cells with MGO, they showed blebs and cell integrity was completely lost in most cases. Although, when coincubating the cells with this 1,2-dicarbonyl and the inhibitor of caspases, cell morphology was greatly recovered, the number of cells displaying the morphology observed in the control cells was increased (Figure 6(d)). It was found that cell viability was significantly recovered upon preincubation with q-VD-OPH and it consequently pointed to apoptosis as the most feasible cell death mechanism produced by MGO (Figure 6(c)).

After that, we used a series of other cell death inhibitors to decipher the cell death mechanism by which cells were dying when incubated with 3-DGal and 3,4-DGE. Hence, we preincubated cells with Ferrostatin-1, an inhibitor of ferroptosis; with 3-MA, an inhibitor of autophagy; and Necrostatin-1, an inhibitor of necroptosis, for 30 minutes, and after that, 3-DGal and 3,4-DGE were added to the cell culture. Cells were incubated with both compounds for 48 hours, and then, cell viability was assayed by trypan blue exclusion. When cells were incubated with 3-DGal and 3,4-DGE, some cells showed irregular borders and blebs. Nevertheless, when cells were coincubated with 1,2-dicarbonyls and cell death inhibitors, no recovery of the cell morphology was noticed (Figure 7(a)). Similarly, when cells were incubated with the 1,2-dicarbonyls and inhibitors of ferroptosis, autophagy, and necroptosis, cell viability was not recovered in any of the assayed conditions (Figure 7(b)).

### 3.6. 3-DGal and 3,4-DGE Activated the Inflammatory Pathways of NF-*κ*B and NLRP3 Inflammasome

Given the impact on cell viability derived from the exposure of the 1,2-dicarbonyl compounds 3,4-DGE, 3-DGal, and 3-DG, and the AGE Pyrr, the subsequent analyses were structured to understand which pathways were underlying the cytotoxicity involved in this reduction of cell viability. The phosphorylation of the IKK*α*/*β* and I*κ*B*α* proteins was evaluated, respectively, on the amino acid residues Ser176/180 and Ser32/36. IKK phosphorylation values are shown as the ratio between the phosphorylated protein and the total protein in the whole protein extract of the samples examined. IKK phosphorylation levels were significantly increased in the 3,4-DGE and 3-DGal treatment groups compared to the control group. Furthermore, these values are comparable to each other. On the other hand, there is no evidence of IKK phosphorylation significantly different from the control group for the samples treated with 3-DG. The consequent phosphorylation of the I*κ*B*α* protein was then evaluated. It can be seen that the observed trend for IKK phosphorylation was comparable to that of I*κ*B*α* phosphorylation. In particular, as regards the parameters related to the phosphorylation both of IKK and of I*κ*B*α*, the phosphorylation appears to be tripled for 3-DGal and slightly more than tripled for 3,4-DGE compared to the control. By analyzing the data related to the 3-DG and Pyrr groups, these are comparable to the control for both parameters. To evaluate the translocation of NF-*κ*B at the nuclear level, the presence of this factor in the cytosolic protein extract and the nuclear protein extract was tested. The results are expressed as the ratio between cytosolic NF-*κ*B and nuclear NF-*κ*B. The results show a significant nuclear translocation of NF-*κ*B in HaCaT cells treated with 3,4-DGE. Nuclear NF-*κ*B is more than five times higher compared to the control. Furthermore, regarding the 3-DGal group, the translocation of NF-*κ*B at the nuclear level can be highlighted. Despite the high standard deviation, it can be seen that the presence of the transcription factor in the nucleus is approximately four times the same in the control group (Figure 8).

Similar results were obtained when the effects on the modulation of the NLRP3 inflammasome pathway were evaluated. As shown in Figure 9, the expression of NLRP3 is more than doubled in the 3,4-DGE and 3-DGal treatment groups compared to the control group. Exactly as observed for the other markers previously examined, the two groups are comparable to each other. However, it should be considered that the exposure concentration of keratinocytes to 3,4-DGE was 10 times lower than that of the exposure to 3-DGal. Following the evaluation of the expression of NLRP3 in the groups under analysis, it was decided to evaluate its activation by searching for the cleaved form of gasdermin-D (GSDMD). NLRP3, once activated, can activate caspase-1 that can cleave (in addition to, for example, the most studied interleukin-1*β*) the GSDMD. The *N*-terminal residue of GSDMD (at 30 kDa) is then able to form transmembrane pores.  Figure 10 also shows the analysis of the inactive form of GSDMD (Pro-GSDMD) and the active form (Activated GSDMD) production in keratinocytes treated with 3-DGal, 3,4-DGE, Pyrr, and 3-DG. The groups exposed to 3,4-DGE and 3-DGal, in addition to causing an increase in the expression of NLRP3 (as seen above), also showed the activation of GSDMD; in these groups of treatment, GSDMD was about five times higher than the inactive form. In contrast, the 3-DG and Pyrr groups did not show any difference in the presence of the two forms compared to the control group.

## 4. Discussion

In the present manuscript, we report for the first time the biological effects that individual glycated amino acids and 1,2-dicarbonyls induce in a keratinocyte cell model. We found that most of the assayed 1,2-dicarbonyls are cytotoxic at a concentration ranging from 50 *μ*mol/L to 500 *μ*mol/L, whereas glycated amino acids do not alter cell viability. Hence, 3-DGal, 3,4-DGE, GO, and MGO highly reduce cell viability. When coincubating the cells with NAC, we found that this antioxidant prevents the decrease in cell viability caused by 1,2-dicarbonyls, which accounts for a possible role of ROS in mediating 1,2-dicarbonyls cytotoxicity. Indeed, we found that 1,2-dicarbonyls increase peroxide, peroxynitrite, and superoxide production in cells, and therefore, the production of SOD1 and SOD2 counters an excessive ROS production. Finally, we found that the 1,2-dicarbonyl MGO leads to cell death by caspase-mediated apoptosis and that 3-DGal and 3,4-DGE activate the NF-*κ*B pathway and drive the activation of NLRP-3 inflammasome, which triggers cell death by pyroptosis.

Up to now, most of the studies that have been published in the field of the biological and pathological roles of AGEs have been conducted using glycated albumin or a mixture of different AGEs to perform the experiments. The procedures used to obtain these substances widely vary from laboratory to laboratory, usually following nonreproducible methodologies, making the results obtained between different research groups hardly comparable. Moreover, AGEs comprise an extensive variety of compounds, with each compound being structurally very different from the other, and thus, they might not exert the same effects in cellular and animal models. In addition to AGEs, albumin glycation produces 1,2 dicarbonyls. Therefore, there is a lack of reproducible methodology, and it is necessary that the role of individual AGEs and 1,2-dicarbonyls should be investigated.

To perform our experiments, the most prevalent glycated amino acids and 1,2-dicarbonyls in foods were synthesized to assay the effects that they might produce individually in cell culture. Since diet is a source of exogenous products of glycation, and the mouth is the first tissue in contact with these compounds, we used an oral mucosa *in vitro* cell model, using the human keratinocyte cell line HaCaT. We found different cytotoxic effects depending on the compound tested. On the one hand, some of the best characterized glycated amino acids, such as CEL and CML, were not cytotoxic in our cell model. As it has been reported, these compounds are present in the plasma of diabetic patients in a concentration up to 1.2 *μ*mol/L for CEL and 2.9 *μ*mol/L for CML and at a concentration up to 1.7 *μ*mol/L and 4.9 *μ*mol/L, respectively, in the plasma in type I diabetes and impaired renal function patients [47]. It has been also reported that plasma CEL/CML concentrations in chronic kidney disease patients are 336 nmol/L and 111 nmol/L, respectively [48]. Moreover, in one study using endothelial progenitor cells, CEL and CML up to a concentration of 4.58 *μ*mol/L and 4.90 *μ*mol/L, respectively, showed no cell toxicity [49]. These concentrations are much lower than our maximum concentration tested, i.e., 1 mol/L, which does not exert any cytotoxic effect triggered by these two glycated amino acids. In the case of MG-H1, its concentration according to several studies in serum of nondiabetic patients is at 76.67 ± 35.93 nmol/L [50] and in plasma at 109.97 ± 46.00 nmol/L [51]. Moreover, the daily intake of CEL was calculated to be ~0.01 mmol, of CML~0.015 mmol, and MG-H1~0.1 mmol. In the case of Pyrr, the intake was estimated to be around 0.08-0.16 mmol [52]. Again, these quantities are below the maximum ones employed in this study, which do not show any harmful effect on our cell model.

Furthermore, we have not found any cytotoxicity of 3-DG in our cellular model, which agrees with another study where this 1,2-dicarbonyl compound was tested in PC12 cells and no cytotoxicity was found [53]. It has been described that the plasma concentration in type 2 diabetes patients of 3-DG is 1.37 *μ*mol/L, of GO 0.74 *μ*mol/L, and of MGO 0.31 *μ*mol/L [54]. In serum of patients with chronic kidney disease, the amounts have been found to be of 1.64 *μ*mol/L for 3-DG, 1.72 *μ*mol/L for GO, and 1.08 *μ*mol/L for MGO [55]. In peritoneal dialysis fluids, 3-DGal has been detected at a concentration of ≤16 *μ*mol/L and 3-DG at a concentration of ≤7 *μ*mol/L [56]. These numbers are below the concentration of these compounds from which we see effects in keratinocytes. However, the concentration of 3,4-DGE in peritoneal dialysis fluids is 9-22 *μ*mol/L [57], which is an amount that already decreases cell viability in our cellular model.

Moreover, some studies using other cell types describe a reduction in cell viability of ~22% with a concentration of 1 mmol/L MGO in leukocytes [58] and 1.6 mmol/L in endothelial cells [59]. MGO is found at high concentrations in Manuka honey [60]. Its cytotoxicity and its mediated NF-*κ*B activation have been reported by several groups [61–63]. Besides, MGO has also been found to increase the phosphorylation of the MAPK family members p-JNK, p-ERK, and p-p38 and highly decrease the levels of MMP-9 and Bcl-2 [64]. MGO has also been associated with metabolism and mitochondrial function, inhibiting glycolysis and mitochondrial complex I [65, 66].

We found that the antioxidant NAC, a synthetic precursor of the intracellular antioxidant glutathione (GSH), can recover cell viability in a different degree upon treatment with 3-DGal, 3,4-DGE, GO, and MGO. This is in accordance with previous studies, which have shown that pretreatment with NAC improved cell viability in MGO-treated cells [67]. Furthermore, in another study, performed this time in the pancreatic beta-cell line INS-1, it was reported that cell viability decreased to 70% when cells were treated for 24 hours with 2 mmol/L MGO. However, this effect was partly recovered when cells were also incubated with 400 *μ*mol/L NAC [68]. It is of notice that the concentration of NAC employed in both studies was much lower than the concentration employed in our study. Moreover, in the first study, the cell culture medium containing NAC was discarded before incubation with MGO. Besides, the concentration of MGO used in the second study in INS-1 cells was much higher than the amount we used. Nevertheless, MGO might produce cytotoxic effects at different concentrations in different cell lines, as shown by other authors [69–73]. The recovery in cell viability upon coincubation with NAC might be due to the capacity of NAC to scavenge free radicals, but it may also be considered that it forms hemithioacetals with MGO in the culture media (Figure 9).

We also saw that cells treated with these 1,2-dicarbonyls produce different ROS, being MGO, which induces a greater production of peroxides and superoxide anion in the cells. Some previous studies have identified an increase in the intracellular levels of ROS after treatment with AGEs [34–36]. They found that glycated human serum albumin, rich in AGEs, induced the expression of E-selectin in the endothelial cells of HUVEC. However, when cells were preincubated with diphenyleneiodonium (DPI), an inhibitor of NADPH oxidase, E-selectin expression was suppressed in a dose-dependent manner. There was indeed an AGEs-induced production of ROS, as it was shown by an increase in 2′,7-dichlorofluorescein (DCF) fluorescence signal upon cell treatment with AGEs [34]. Similar results have been reported in a cellular model of macrophages. When these cells were treated with the product of the reaction between MGO and bovine serum albumin, rich in MGO-derived AGEs, ROS production assayed by 2′,7′-dichlorofluorescein diacetate (DCFH-DA) was increased. The origin of these ROS might be NADPH oxidase since, upon incubation with AGEs, the mRNA of NOX1 and NOX2 was highly increased. Moreover, ROS-mediated damage to proteins, measured as protein carbonyls and advanced oxidation protein products (AOPPs), was raised as well upon incubation with AGEs. Interestingly, coincubation with pterostilbene, a plant polyphenol with antioxidant properties, decreased ROS production, NOX1 and NOX2 expression, and oxidative damage to proteins [36]. A recent study performed in human endothelial cells showed that when cells were incubated with glycated albumin, it was induced an increase in the concentration of H_2_O_2_, O_2_^•-^, and ^•^NO as well as an increase in CAT, GPX, and SOD1 activities and AOPPs production. The source of these AGEs-induced ROS proved to be the mitochondria and NADPH oxidases as tested employing myxothiazol, an inhibitor of complex III of mitochondria, and the NADPH oxidase inhibitor, apocynin. Furthermore, coincubation with a plant extract with a high polyphenol content reduced the AGEs-mediated ROS production in this cellular model [35]. Nevertheless, all of these studies employed glycated albumin as a source of AGEs, and they did not demonstrate the effect of individual compounds, while in our study, we confirm that the molecules producing cytotoxic effects in our cellular model are indeed 1,2-dicarbonyls.

In recent studies, it has been found that MGO also induces ROS production in human embryonic kidney cells [74]. In SH-SY5Y cells, it was reported an increase in H_2_O_2_, O_2_^•-^, and ^•^NO production after incubating with MGO, which also induced lipid peroxidation, protein carbonyls and thiols, protein nitration, and DNA oxidative damage. Besides, all of these effects were partly reversed by incubation with antioxidants [75]. However, all in vitro studies where the role of single 1,2-dicarbonyls is investigated are performed employing MGO, and here, we show for the first time an increased production of ROS by 3-DGal, 3,4-DGE, and GO.

It is already studied that AGEs can produce cell death, being the apoptosis proposed mechanism in the majority of cases. However, in this work, we show that, when assayed individually, not all of the compounds exert the same effect. Indeed, we show that MGO induces apoptosis in our cellular model, as assayed using Annexin-V staining and an inhibitor of apoptosis. This is in agreement with some recently published works where they show apoptotic death following treatment with MGO [58, 76]. Nevertheless, when we assayed 3-DGal and 3,4-DGE, we found that, surprisingly, both 1,2-dicarbonyls do not enhance apoptosis in the cells. Moreover, keratinocytes exposed to 3-DGal and 3,4-DGE in the presence of inhibitors of death by autophagy, ferroptosis, and necroptosis were not able to preserve from death. Interestingly, these compounds were able to induce the activation of gasdermin, the protein that triggers pyroptosis, one form of programed necrosis. Thus, we propose here that ROS produced by 3-DGal and 3,4-DGE promote pyroptosis through NLRP-3 inflammasome activation [77, 78], leading to gasdermin cleavage, following formation of pores in the membrane of the cell and, thus, swelling and membrane rupture [79].

It has already been described that AGEs, by interaction with their receptor RAGE, initiate several signal transduction cascades such as NF-*κ*B, which ultimately lead to the promotion of inflammation or apoptosis, since they produce cytokines, chemokines, and some proinflammatory molecules [18, 23, 37, 80]. In this study, we show how 3-DGal and 3,4-DGE individually activate the NF-*κ*B pathway for the first time. The analysis shows a significant translocation of the factor NF-*κ*B at the nuclear level after 3,4-DGE and 3-DGal treatment. The translocation of NF-*κ*B causes an increased expression of the NLRP3 inflammasome. NLRP3 inflammasome appears to be overexpressed and activated after incubation with 3,4-DGE and 3-DGal. The activation of the NLRP3 inflammasome is confirmed by the presence of the *N*-terminal residue of GSDMD. After oligomerization, the *N*-terminal residue of GSDMD inserts itself into the membrane, generating the transmembrane pores responsible for pyroptotic cell death. Pyroptosis may be the ROS-dependent cell death mechanism implicated in reducing viability in keratinocytes exposed to 3,4-DGE and 3-DGal.

3,4-DGE is a dehydration product of 3-DG and 3-DGal, and it is the most cytotoxic compound examined in this study. 3,4-DGE contains a, *β*,*γ*-unsaturated *α*-dicarbonyl structure, which can undergo the Michael reaction in addition to the direct reaction of the carbonyl groups. Michael reaction of 3,4-DGE with glutathione (GSH) leads to an irreversible adduct due to the depletion of GSH itself with a consequent increase in oxidative stress [81], which causes the activation of the detected signal pathways. It is interesting to note that the signaling pathway activated by 3-DGal also appear to be the same activated by 3,4-DGE, although to have this comparable effect 3-DGal must be administered at a concentration 10 times higher than 3,4-DGE. Therefore, it is proposed that 3-DGal cytotoxicity is due to facile dehydration of the compound to 3,4-DGE, which may be the actual cytotoxic form. Furthermore, it should be noted that 3-DGal, but not its epimer 3-DG, can give such effects. The reason that 3-DG and 3-DGal exhibit two different cytotoxic behaviors may reside in the kinetics of dehydration to give 3,4-DGE. In a literature report, the formation of 3,4-DGE from 3-DGal was observed to be faster than from 3-DG [82].

Finally, it is worth mentioning that the bioavailability of these compounds might vary, given their chemical differences. Membrane solubility, the presence of compound transporters, or perhaps the identification of receptor-mediated signaling pathways in the toxicological profile of AGEs and 1,2-dicarbonyls should be further investigated.

## 5. Conclusion

Isolated glycated amino acids and 1,2-dicarbonyls do not deliver the same biological effect in human epithelial cells. ROS production and cell death are mechanisms of cytotoxicity derived from 1,2-dicarbonyls.

## Figures and Tables

**Figure 1:** Chemical structures of the compounds tested in the present study. CML: N-*ε*-carboxymethyllysine; CEL: N-*ε*-carboxyethyllysine; Pyrr: pyrraline; MG-H1: methylglyoxal-derived hydroimidazolone 1; GO: glyoxal; MGO: methylglyoxal; 3-DG: 3-deoxyglucosone; 3,4-DGE: 3,4-dideoxyglucosone-3-ene; 3-DGal: 3-deoxygalactosone.

**Figure 2:** Effect of individual 1,2-dicarbonyls and glycated amino acids on cell viability. (a) Cell viability upon incubation with individual 1,2-dicarbonyls. (b) Cell viability upon incubation with 3,4-DGE. (c) Cell viability upon incubation with individual glycated amino acids. Results are expressed as mean ± SEM (*n* = 6). ^∗^*p* < 0.05*vs*. CON, ^∗∗^*p* < 0.01*vs*. CON, ^∗∗∗^*p* < 0.001*vs*. CON.

**Figure 3:** Effect of individual 1,2-dicarbonyls on cell cycle. (a) Propidium iodide fluorescence was measured by flow cytometry. One representative experiment is shown. (b) Cell population percentage in each stage of cell cycle. Here, cell treatments consisted of 750 *μ*M 3-DGal, 75 *μ*M 3,4-DGE, 1 mM GO, and 500 *μ*M MGO. Results are expressed as mean ± SEM (*n* = 3). ^∗∗^*p* < 0.01*vs*. CON, ^∗∗∗^*p* < 0.001*vs*. CON.

**Figure 4:** Cell viability recovery after coincubation with 1,2-dicarbonyls and NAC. (a) A representative micrograph for each condition is shown. For each condition, micrographs shown in the first row were taken at 100x original magnification, and micrographs in the second row were taken at 400x original magnification. Arrows indicate blebs. (b) Cell viability upon coincubation with 3-DGal and NAC. (c) Cell viability upon coincubation with 3,4-DGE and NAC. (d) Cell viability upon coincubation with GO and NAC. (e) Cell viability upon coincubation with MGO and NAC. Results are expressed as mean ± SEM (*n* = 3). ^∗^*p* < 0.05*vs*. CON, ^∗∗^*p* < 0.01*vs*. CON, ^∗∗∗^*p* < 0.001*vs*. CON, ^##^*p* < 0.01*vs*. no 1,2-dicarbonyl, ^###^*p* < 0.001*vs*. no 1,2-dicarbonyl.

**Figure 5:** Free radical and antioxidant enzymes production upon application of 1,2-dicarbonyls. (a) Production of peroxide and peroxynitrite as measured by DHR fluorescence intensity. (b) Production of superoxide as measured by DHE fluorescence intensity. (c) Production of mitochondrial superoxide as measures by MitoSOX fluorescence intensity. (d) Representative western blot experiment. (e) Production of SOD1 as analyzed by quantification of western blot optical density. (f) Production of SOD2 as analyzed by quantification of western blot optical density. (g) Production of catalase as analyzed by quantification of western blot optical density. (h) Ratio between the production of SOD2 and catalase. Arbitrary 1.0 value was given to the WT group. Here, cell treatments consisted of 750 *μ*M 3-DGal, 75 *μ*M 3,4-DGE, 1 mM GO, and 500 *μ*M MGO. Results are expressed as mean ± SEM (*n* = 3). ^∗^*p* < 0.05*vs*. CON, ^∗∗^*p* < 0.01*vs*. CON, ^∗∗∗^*p* < 0.001*vs*. CON.

**Figure 6:** Cell death by apoptosis after incubation with 1,2-dicarbonyls. (a) Annexin-V and 7-AAD fluorescence was measured by flow cytometry. One representative experiment is shown. (b) Percentage of apoptotic cells in the cell culture. Positive cells for Annexin V and for both Annexin V and 7-AAD were considered apoptotic. (c) Cell viability upon coincubation with MGO and the apoptosis inhibitor Q-VD-OPh. (d) Cell viability recovers after coincubation with apoptosis inhibitor Q-VD-OPh. A representative micrograph for each condition is shown. For each condition, micrographs shown in the first row were taken at 100x original magnification, and micrographs in the second row were taken at 400x original magnification. Arrows indicate blebs. Here, cell treatments consisted of 1 mM 3-DG, 750 *μ*M 3-DGal, 75 *μ*M 3,4-DGE, 1 mM GO, and 500 *μ*M MGO. Results are expressed as mean ± SEM (*n* = 3). ^∗∗∗^*p* < 0.001*vs*. CON, ^###^*p* < 0.001*vs*. no 1,2-dicarbonyl.

**Figure 7:** Cell viability recovery after coincubation with cell death inhibitors. (a) A representative micrograph for each condition is shown. For each condition, micrographs shown in the first row were taken at 100x original magnification, and micrographs in the second row were taken at 400x original magnification. Arrows indicate blebs. (b) Cell viability upon coincubation with the ferroptosis inhibitor Ferrostatin-1. (c) Cell viability upon coincubation with the autophagy inhibitor 3-MA. (d) Cell viability upon coincubation with the necroptosis inhibitor Necrostatin-1. Here, cell treatments consisted of 750 *μ*M 3-DGal and 75 *μ*M 3,4-DGE. Results are expressed as mean ± SEM (*n* = 3). ^#^*p* < 0.05*vs*. no 1,2-dicarbonyl, ^##^*p* < 0.01*vs*. no 1,2-dicarbonyl.

**Figure 8:** Activation of the NF-*κ*B pathway upon incubation with 1,2-dicarbonyls. (a) IKK*αβ* phosphorylation. A representative western-blot experiment is shown. Graphic represents the ratio between the production of p-IKK*αβ* and total IKK*αβ* as analyzed by quantification of western blot optical density. (b) I*κ*B phosphorylation. A representative western blot experiment is shown. Graphic represents the ratio between the production of I*κ*B and total I*κ*B as analyzed by quantification of western blot optical density. (c) NF-*κ*B activation. A representative western blot experiment is shown. Graphic represents the ratio between the production of nuclear p65 NF-*κ*B and cytosolic NF-*κ*B as analyzed by quantification of western blot optical density. Arbitrary 1.0 value was given to the CON group. Here, cell treatments consisted of 750 *μ*M 3-DGal, 75 *μ*M 3,4-DGE, 1 mM Pyrr, and 1 mM 3-DG. Results are expressed as mean ± SEM (*n* = 3). ^∗^*p* < 0.05*vs*. CON, ^∗∗^*p* < 0.01*vs*. CON, ^∗∗∗^*p* < 0.001*vs*. CON.

**Figure 9:** Reaction of N-acetylcysteine with MGO under formation of a hemithioacetal.

**Figure 10:** NLRP3 inflammasome and gasdermin activation upon incubation with 1,2-dicarbonyls. (a) NLRP3 inflammasome activation. A representative western blot experiment is shown. Graphic represents the production of NLRP3 as analyzed by quantification of western-blot optical density. (b) Gasdermin activation. A representative western blot experiment is shown. Graphic represents the production of progasdermin and activated gasdermin as analyzed by quantification of western blot optical density. Arbitrary 1.0 value was given to the CON group. Here, cell treatments consisted of 750 *μ*M 3-DGal, 75 *μ*M 3,4-DGE, 1 mM Pyrr, and 1 mM 3-DG. Results are expressed as mean ± SEM (*n* = 3). ^∗^*p* < 0.05*vs*. CON, ^∗∗^*p* < 0.01*vs*. CON, ^∗∗∗^*p* < 0.001*vs*. CON, ^##^*p* < 0.01*vs*. progasdermin.

## Data Availability

The data used to support the conclusions of this study are available from the corresponding authors upon request.

## Abbreviations

3,4-DGE: 3,4-Dideoxyglucosone-3-ene
3-DG: 3-Deoxyglucosone
3-DGal: 3-Deoxygalactosone
7-AAD: 7-Aminoactinomycin D
AGEs: Advanced glycation end products
AOPPs: Advanced oxidation protein products
Bcl-2: B-cell lymphoma 2
BSA: Bovine serum albumin
CAT: Catalase
CEL: N-*ε*-(carboxyethyl)lysine
CML: N-*ε*-(carboxymethyl)lysine
DCF: 2′,7-Dichlorofluorescein
DCFH-DA: 2′,7′-Dichlorofluorescein diacetate
DHE: Dihydroethidium
DHR-123: Dihydrorhodamine 123
DMEM: Dulbecco's modified Eagle's medium
DMSO: Dimethyl sulfoxide
DPI: Diphenyleneiodonium
EDTA: Ethylenediaminetetraacetic acid
ERK1/2: Extracellular signal-regulated kinase 1/2
FITC: Fluorescein isothiocyanate
GO: Glyoxal
GPX: Glutathiones peroxidase
GSDMD: Gasdermin-D
GSH: Glutathione
HRP: Horseradish peroxidase
HUVEC: Human umbilical vein endothelial cells
I*κ*B*α*: Nuclear factor of kappa light polypeptide gene enhancer in B-cells inhibitor alpha
IgG: Immunoglobulin G
IKK*β*: Inhibitor of nuclear factor kappa-B kinase subunit beta
MAPK: Mitogen-activated protein kinases
MG-H1: Methylglyoxal-derived hydroimidazolone-1
MGO: Methylglyoxal
MMP-9: Matrix metalloproteinase 9
MTT: 3-(4,5-Dimethylthiazol-2-yl)-2,5-diphenyltetrazolium bromide
NAC: N-acetyl-cysteine
NADPH: Nicotinamide adenine dinucleotide phosphate
NF-*κ*B: Nuclear factor kappa-light-chain-enhancer of activated B cells
NLRP3: NOD-, LRR-, and pyrin domain-containing protein 3
NOX1: NADPH oxidase 1
NOX2: NADPH oxidase 1
PAGE: Polyacrylamide gel electrophoresis
PBS: Phosphate-buffered saline
PI: Propidium iodide
PI3K: Phosphatidylinositol 3-kinase
PVDF: Polyvinylidene difluoride
Pyrr: Pyrraline
Q-VD-OPh: Quinoline-Val-Asp-Difluorophenoxymethyl Ketone
RAGE: Receptor for AGEs
RNase: Ribonuclease
ROS: Reactive oxygen species
SOD1: Superoxide dismutase 1
SOD2: Superoxide dismutase 2
TBS-T: Tris-buffered saline with 0.1% Tween ® 20 Detergent.
